# Analysis of the Influence of Human Resources on the Economic Development of Minority Areas Based on Data Mining

This article has been retracted.

**DOI:** 10.1155/2022/8147537

**Published:** 2022-10-12

**Authors:** Qian Guo, Yubo Liu, Changde Zheng

**Affiliations:** Institute of Western China Economic Research, Southwest Minzu University, Chengdu, Sichuan 610041, China

## Abstract

In order to break the bottleneck of the human capital stock restricting local economic growth in the typical western regions with backward national economic development, a research on the analysis of the impact of human resources on the economic development of ethnic regions based on data mining is proposed. On the basis of systematically reviewing the current situation and the theoretical basis of the relationship between human capital and economic growth, the method of combining normative research and empirical research is adopted, and the theories of macroeconomics, development economics, and regional economics are synthesized. In the research, the human capital and economic development in a certain western region are analyzed by establishing an econometric model. The results show that the average value of each year is taken as the inspection index, and the contribution rate is 0.0012, which shows that the contribution of human capital stock in economic growth is very small, indicating that physical capital stock is still the main driving force for local economic development. It is concluded that the research provides some relevant recommendations for human capital development to achieve sustainable local economic development.

## 1. Introduction

Historical materialism believes that the mode of production is the decisive force for social development, determines the development and change of a society, and determines the transformation of a society from one form to another [1]. The mode of production includes two aspects: productivity and production relations. These two aspects are in a contradictory movement from adaptation to incompatibility and then to new adaptation and incompatibility, in a cycle that promotes social development. In this contradictory movement, laborers are the ultimate driving force. The best among the laborers' talents are the most active and revolutionary factors in the mode of production and the driving force and source of social development and progress. Among the many resources that promote social development and progress, human resources are of decisive significance. Therefore, the development and utilization of human resources are worth studying.

From an international background, countries around the world generally attach importance to the research and practice of the development and utilization of human resources. Since the 20th century, the general attention of countries around the world has been mainly based on the following reasons. First, with the improvement of social productivity and the rapid increase of the global population, natural resources are becoming increasingly withered and the ecological environment is deteriorating. Second, the fact that the economies of countries and regions with poor natural resources can develop rapidly shows that modern science and technology, especially high-quality talents, have played a key role. Third, the rapid development and application of science and technology have greatly improved the living standards of human beings and also made human work more and more specialized and mechanized, and labor intensity and pressure have increased. At the same time, it also inhibits people's enthusiasm for work and restricts the full development of talents and the full exploration of potential. Therefore, more and more attention has been paid to the development and utilization of human resources, especially human resources [2]. Fourth, with the rapid economic development, people's ideas are also undergoing fundamental changes. The great social and economic development has improved people's material living conditions and levels as a whole, and at the same time has caused profound changes in people's ideas. How to create system and mechanism conditions and build a career platform for the all-round development of talents is a major issue facing today's society. Fifth, economic globalization has entered a new stage, and the degree of economic competition is increasing day by day. The rise of the third and fourth scientific and technological industrial revolutions not only highlights the importance of human resources but also shows that the competition in the economic field between countries and ethnic groups is essentially the competition of talents, which is the development and utilization of human resources. At present, many countries in the world have set off a fierce and even almost crazy competition for talents and have successively established institutions for the development and utilization of human resources.

From the theoretical point of view, although there are some achievements in the development and utilization of human resources in the extremely poor areas of ethnic minorities, the achievements are only a small amount. Even if it has certain regional characteristics, it is not general [3]. Judging from the actual situation in the extremely poor areas of ethnic minorities, attention must be paid to the development and utilization of human resources. The great cause of the development of ethnic minority poverty-stricken areas has created a favorable environment for the all-round development of the people in ethnic minority poverty-stricken areas and has also provided a broad stage for the development and utilization of human resources in ethnic minority poverty-stricken areas. However, the competition between technology and talents is becoming more and more fierce, and the status and role of talents in economic development are becoming more and more important. The problem of talent flow being restricted by economic conditions, the natural environment, and policy orientation is becoming more and more prominent. How to win the initiative in this increasingly fierce competition for talents and how to develop and make good use of human resources is a major issue that needs to be solved urgently in the impoverished areas of ethnic minorities. Therefore, it is necessary to base the development and utilization of human resources in the poverty-stricken areas of ethnic minorities under the background of the theory of human resources and conduct in-depth explorations according to the particularities of the development and utilization of human resources in the poverty-stricken areas of ethnic minorities, as shown in Figure 1.

## 2. Literature Review

At present, most scholars' research basically only reflects the influence and function of a single factor on the economic development of ethnic areas and has also achieved relevant results. Cunha et al. proposed in the study of the economic development of Qinghai Province in western China, starting from the necessity of developing the national cultural industry, how to use the cultural industry to rapidly develop the local economy and alleviate ethnic conflicts in the areas with diverse ethnic groups and a lack of natural resources was analyzed [4]. Purkayastha et al. put forward how to use the principle of multiethnic economic symbiosis to achieve sustainable and coordinated economic development in multiethnic areas under the new normal in the issue of the development of the Tibet-Yi Corridor [5]. Ksaa pointed out that to build an external driving force mechanism for the independent economic development of ethnic autonomous regions, FDI (foreign trade, foreign direct investment) should be actively introduced and effectively utilized to promote stable economic growth [6]. Ly et al. clearly pointed out that human capital is an important element of social and economic development and the fundamental driving force for economic development in underdeveloped ethnic areas [7]. Wesemann pointed out in the research on the economic and social development of Inner Mongolia that ecological civilization is the driving force for promoting the economic development of ethnic minority areas, and the great achievements in ecological construction provide an ecological guarantee for economic and social development and are the important foundation of the sustainable development of the economy and society [8].

Regional economic development requires power to obtain further development. In this process, strengthening research on power systems can provide necessary conditions for regional economic development. In the process of regional economic development, continuous and efficient innovation activities can reduce the cost of the regional economy, improve the efficiency, and promote the steady development of the regional economy. If there is no driving force for regional economic development, there is no supporting force, lifting force, guiding force, centripetal force, or system synergy and there will be no development force, let alone vitality. According to the principle of general system theory, from the perspective of the operation of a circular economy, Adesina, Ksaa believed that ecological power came from external environmental pressure, internal interest pressure, and market competition pressure, which is reflected in the response, trade-off, and control of regional subjects to these three pressures. The ecological dynamic system should be constructed according to the model of ecological pressure-system structure-system function,” so as to promote the “social-economic-environment” system to embark on a benign development path from mutual isolation to gradual integration [6].

In terms of national economy, on the basis of the status quo of Baise's economic development, Yang et al. proposed that it is necessary to improve the dynamic system of the economic development of frontier central cities. The complex relationship between ethnic groups and religions brings about a lack of innovation power for regional economic development. To this end, it is necessary to make up for the lack of power by striving to realize the internalization effect of external power, mining traditional national cultural and political resources, strengthening the growth of internal power, and promoting the aggregation of internal and external power with effective measures [9]. Chao et al. proposed that this market-controlled economy, which turns labor, natural resources, and capital into commodities, will lead to many collisions and cancellations for all peoples and societies around the world. Factors keep growing. Therefore, the economic formation is inevitably controlled by the socially controlled economic formation. It is believed that this is a social and cultural law that works for all nations and societies [10]. Santoso found that the development of modernization will have a huge impact on the traditional social structure. In a multicultural society, the performance of this shock will be different [11]. Yin and Choi regarded Chinese culture as a unity of diversity. He believed that such a “multiple unity” was developed in a long-term historical process and proposed cultural self-consciousness. He conducted numerous social and historical surveys of ethnic minorities and put forward the theories of ”small town construction,” “township enterprises,” “Southern Jiangsu model,” and “Wenzhou model” [12].

In the research, the status quo of human resource development in ethnic areas and its restrictive factors are first analyzed. At present, the characteristics of human resources in ethnic areas of our country are low population quality, small total amount, and unreasonable structure. Due to the constraints of ideological conditions, capital and infrastructure, and social systems in ethnic areas, the development of human resources has been severely restricted. The physical capital stock and human capital stock are estimated for a certain ethnic region, and the relationship between human capital and economic growth in this region is empirically analyzed by using the selected model.

## 3. Research Methods

### 3.1. Status Quo of Human Resource Development in Minority Areas

Generally speaking, the human resources situation in ethnic areas is low population quality, the small total amount of talents, unreasonable distribution, low level of talent, and unreasonable structure.

#### 3.1.1. The Quality of Population in Ethnic Areas Is not High

First, the health quality of the population in ethnic areas is low. Due to the backward economic environment in ethnic areas, a relatively complete healthcare system has not been established, so people's health status is generally poor [13]. On the one hand, economic conditions do not allow people to pay more attention to their own health status, and there is no money for treatment. The methods of “exorcising evil spirits” and “worshiping gods” are all reasons for the poor health of the population in the region.

Second, the population in ethnic areas is low in education. The poverty of ethnic minority areas in our country makes the educational level of the population in these areas generally relatively low, which greatly increases the difficulty of realizing industrialization in ethnic minority areas. The illiteracy and semiliteracy rate in ethnic areas is 27.2%, which is higher than the national average of 23.2%. The proportion of the population with high school, junior college, and above education in the total population is also significantly lower than the national average, and the average years of education is also relatively low. See Table 1 for details.

Finally, there are few scientific and technological practitioners in ethnic areas. Technological practitioners mainly refer to practitioners in various institutions engaged in scientific and technological research and development. These institutions include universities, government research institutes, and corporate research institutions, as well as grassroots institutions engaged in technology promotion. In the western region, where ethnic minorities are densely populated, there are only 3.3 scientific and technological personnel per 10,000 people on average, compared with 5.6 scientific and technological personnel per 10,000 people in the eastern region and 3.6 scientific and technological personnel in the whole country [14]. At the same time, the number of scientific and technological personnel engaged in humanities and social sciences in the western region is even lower, with an average of only 0.09 researchers in social and humanities per 10,000 people, compared with 0.18 in the eastern region and 0.11 in the whole country. This shows that the humanities and social sciences in the western region are still quite backward, and the overall thinking in the western region is still relatively conservative.

Most of the ethnic areas exist in the west. Through the analysis of the total amount and distribution of talents in the west, the relevant situation of the ethnic areas can be briefly understood. By 2021, the total number of talents in the western region will be about 11.48 million, accounting for about 19% of the national total. The number of civil servants is 2.04 million, accounting for about 17% of the total talent in the western region. There are about 7.61 million professional and technical talents, accounting for about 66% of the total talents in the western region. There are about 1.61 million ethnic minority talents, accounting for 14% of the total number of talents in the western region. This shows that there is a shortage of talents in ethnic areas. Compared with many other factors, talents are often more difficult to obtain. The lack of human resources has become a key factor restricting the development of the industrial economy in ethnic areas.

By analyzing the distribution of talents in the western region, the distribution of talents in ethnic regions can be obtained. The unreasonable distribution of talents in the western region is reflected in the unreasonable geographical distribution and the unreasonable distribution of departments. First, the unreasonable geographical distribution is analyzed [15]. Talents are concentrated in regions with relatively developed regional economies, which means the western region, where the overall talent is lacking, has a relative surplus of talents, while the vast underdeveloped areas do not have the talent available. For example, 80% of the talents in Qinghai Province is concentrated in Xining City. 88% of the talents in the affiliated provinces is concentrated in Lanzhou City. The total amount of talents in Chengdu City, Sichuan Province, is much larger than the total amount of talents in the three prefectures of Ganzi, Aba, and Liangshan combined. The second is the unreasonable distribution of departments. Most talents in the western region are concentrated in state-owned enterprises and institutions [16]. The proportion of talented people engaged in secondary industry is relatively low, which is obviously not conducive to the development of the industrial economy in ethnic areas. See Table 2 and Figures 2–4 for details.

#### 3.1.2. The Talent Level in Ethnic Areas Is Low and the Structure Is Unreasonable

The level of talents in the western region is relatively low, and there is a lack of high-level talents, and the proportion of highly educated talents in the total talents is relatively low. Judging from the professional titles held by state-owned professional and technical personnel, the proportion of talents with intermediate and senior professional titles is obviously low. See Tables 3 and 4 for details. Considering the education situation in ethnic areas, the level of talents in ethnic areas is even less optimistic.

### 3.2. Factors Restricting Human Resource Development in Minority Areas

#### 3.2.1. Constraints of Ideological Conditions

Ethnic areas are generally located in remote areas of the motherland. Due to the combined effect of various factors such as geography and humanities, ethnic areas are relatively closed and have poor acceptance of new things. Many ethnic areas are still in an agricultural society, and “one cow per 20 acres of land, and the wife and children are on the head of a Kang” is the standard for a happy life. The masses cannot see the outside world and are always enclosed in a low-level, low-standard circle [17].

There is a phenomenon of “poor culture” in ethnic areas. “Poverty culture” refers to the idea of “letting fate” which often exists in poor areas and taking no action against the local reality of poverty. At the same time, it also refers to the thought of “waiting, relying on, and wanting.” Many people, even some cadres, regard the aid of superiors as an infinite resource and focus their energy on securing aid from superiors, rather than relying on their own strength to develop the local economy. This kind of thinking has caused the problem that the antipoverty rate in ethnic areas remains high, “the poverty alleviation year by year.”

It can be seen that fundamentally changing the ideological concept of people in ethnic areas being backward and ignorant is the fundamental guarantee for the smooth development of human resources in ethnic areas.

#### 3.2.2. Constraints on Capital and Infrastructure

The economic development of many ethnic areas is relatively backward, and the local governments have insufficient financial resources. Many local governments can only maintain basic office operations and are unable to provide financial guarantees for human resource training [18]. Insufficient financial resources make the investment in scientific and technological research and development and per capita education funds in ethnic areas insufficient. For example, the R&D expenditure in the eastern region accounts for 0.67% of the total regional GDP, while the data in the western region is only 0.394%.

At the same time, the shortage of funds also limits investment in infrastructure. This is first manifested in the poor medical and health conditions in ethnic areas. Many areas, especially rural areas, lack basic medical structures [19]. It has seriously affected the health of the local people. According to the fourth national census, life expectancy in Qinghai is 8.0 years lower than the national average, and life expectancy in Xinjiang is 6.0 years lower than the national average. Secondly, in terms of the quality of life of residents, such as the quality of drinking water, housing quality, etc., the situation in ethnic areas is not satisfactory.

The low level of capital investment also caused problems in the information exchange between ethnic areas and the outside world [20–23]. In today's information age, a large part of the people in ethnic areas have not had access to computers and the Internet, and the coverage of radio and television is also very low. The difficulty of information exchange also makes the human resources in ethnic areas not well circulated. It seriously affects the allocation of human resources, and the problem of talent waste is very prominent.

#### 3.2.3. Constraints of the Social System

Minority areas are areas where the process of institutional reform in our country is relatively slow [24, 25]. A large number of state-owned enterprises and institutions have gathered a large number of talents in ethnic areas. The talents of these units cannot go up and down, and they can enter but not go out. The egalitarian ideology of “big pot of rice” and “golden rice bowl” is more serious, lacking incentives and crisis awareness. The enterprise lacks vitality, the economic benefit is poor, and the operational efficiency of the institution is low. They are not motivated to develop their own human resources and strengthen their competitiveness.

Today, when mental work is becoming more and more valuable, the value created by mental workers is increasing. Therefore, it is a matter of course that they should be paid relatively high. In ethnic areas, there is no corresponding reward mechanism, and material rewards for high-level talents are insufficient. On the one hand, this has resulted in the weakening and shortage of talent creativity, and on the other hand, the phenomenon of the outflow of high-quality talents has become more and more severe.

### 3.3. The Impact of Human Capital on Economic Growth in a Region

#### 3.3.1. Model Establishment

In order to more accurately calculate the contribution of human capital to economic growth in a certain region in western country, based on Solow's total production function method, an economic growth model is constructed [26–29]. In order to establish a model that can further reflect the impact of human capital on economic growth, on the basis of the Cobb-Douglas production function model on the relationship between output and input labor and capital, taking into account the production function of human capital, the level of human capital is introduced to establish a relationship between human capital in a certain region and economic growth. The model of the endogenous effect is the following formula:

(1) $$\begin{array}{c} Y=AL^{\alpha }K^{\beta }H^{\lambda }\text{.} \end{array}$$

In the Cobb–Douglas production function, the following assumptions exist. (1) The level of production technology and factor prices remain unchanged. (2) The returns to scale remain unchanged, that is, the proportion of output increases is equal to the proportion of various production factors. (3) Capital and labor classes substitute for each other. Both capital and labor have diminishing marginal returns. The model established in the research also has the above assumptions, in which technological progress is regarded as an unchanged constant *A*, and the other variables have the following meanings. *Y* is output, expressed by regional GDP. L is the amount of labor force, *K* is the physical capital, and H is the level of human capital, which in the research is the number of years of education per capita. *α*, *β*, and *λ* are the output contribution of manual labor input, the output contribution of physical capital input, and the output contribution of human capital input, respectively. In the Cobb–Douglas production function, *α*+*β* represents the return to scale, and in this model, *α*+*β*+*λ* also represents the return to scale. Moreover, according to the new growth theory, due to the increasing return of human capital investment, the return to scale *α*+*β*+*λ* calculated in the research should be greater. The model not only fully considers the production function of human capital but also fully considers the external effect of human capital on other nonhuman capital factors, which can accurately reflect the functional relationship between input factors and output, so as to accurately judge the role of human capital in economic growth.

Taking the logarithm of both sides of the above formula, the following formula can be obtained:

(2) $$\begin{array}{c} \ln\;Y=\ln\;A+\alpha \;\ln\;K+\beta \;\ln\;L+\lambda \;\ln\;H\text{.} \end{array}$$

The following will build a regression model with this function for analysis.

#### 3.3.2. Data Selection and Processing

The data required in the research are as follows: ① the GDP of a certain region, that is, a certain region; ② the number of labor force in a certain region; ③ the stock of physical capital in a certain region; and ④ the human capital of a certain region.

*(1) Gross Domestic Product of a Certain Region (Y)*. The gross domestic product of a certain region refers to the total value of the final products and services produced and provided in a certain period of time within the entire scope of a certain region [30–32]. Since each year is calculated at the price of the current year, in order to eliminate the influence of price changes, here the revised real with the year is used as the base period. The conversion formula is as follows:

(3) $$\begin{array}{c} Actual\;{GDP}_{t}=\frac{Nominal\;{GDP}_{t}^{*}GPI\left(1978=100\right)}{{CPI}_{t}}\text{.} \end{array}$$

In formula (3), the actual represents the GDP after conversion in the t-th year, with 1978 as the base period. The nominal GDP_*t*_ represents the GDP calculated at the actual price of the year. GPI(1978=100) represents the consumer price index with 1978 as the base period. CPI_*t*_ represents the consumer price index of the current year. The actual data of each year in a certain region after conversion are shown in Table 5.

*(2) Number of Labor Force (L)*. The number of labor force referred to here is the number of laborers in the whole society in a certain region, that is, the number of employees. In some research studies, it is believed that there may be considerable overlap between the labor input and the human capital input, which affects the accuracy of the analysis and therefore separates the two. Here, it is believed that the impact of this error is small, and the number of workers is still used to establish the measurement model.

*(3) Capital Stock (K)*. Data on physical capital stocks are harder to come by. Physical capital stock has no ready-made time series data and can only be roughly estimated based on relevant indicators [33]. Among the various methods for measuring capital stock, the most commonly used estimation method is the “perpetual inventory method.” This method requires selecting a year with relatively complete stock data as the basis. According to the new investment in each period and the depreciation rate of various assets, the capital stock of the entire investigation period can be obtained by forward or backward recursion.

For the “perpetual inventory method,” it is believed that the capital stock can be obtained from the following formula:

(4) $$\begin{array}{c} K_{t}=I_{t}+\left(1-A_{t}\right)K_{t-1}\text{.} \end{array}$$

In formula (4), *K*_*t*_ is the capital stock in year *t*, *I*_*t*_ is the total investment in year *t*, *A*_*t*_is the depreciation rate in year *t*, and K_t−1_is the capital stock in year *t* − 1. As mentioned above, it can be seen that this is a recursive method, and the existing methods of capital stock research are basically carried out on this basis. There is a big difference. The physical capital stock values for each year in the region are shown in Table 6.

*(4) Human Capital Measurement*. The method used in the research to measure human capital is the years of the education method. To measure with this method, data on human capital stock, illiterate and semiilliterate population, primary school education level, junior high school level education level, high school education level population, and college education level population are needed in the region [34–36]. Considering that there are few data in this region, and the data are only available in individual years, the data of the province are used to process, and the measure of human capital in the region is obtained based on the data of the province, except for a specific proportion.

First, the years of education method is used to estimate the human capital stock of employees in the province.

 
*H*_1_is the illiterate (the population aged 15 years and above who are illiterate and seldom literate), the average years of education are used in the research as years.
 
*H*_2_ is primary school education, mainly based on ordinary primary school education. At present, the school system of ordinary primary schools in our country is years, and the average years of education are used in the research.
 
*H*_3_ is the education level of junior high school, mainly based on ordinary junior high school.
 
*H*_4_ is high school education level, which covers ordinary high schools, secondary professional and technical schools, vocational high schools, and technical schools, etc. The research is calculated by per capita years of education.
 
*H*_5_ is a college degree or above, and the research is calculated by per capita education years.

Therefore, the calculation formula of human capital stock is shown as formulas (5) and (6).

(5) $$\begin{array}{c} Human\;capital\;stock\;H=1*H_{1}+6*H_{2}+9*H_{3}+12*H_{4}+16*H_{5,} \end{array}$$

(6) $$\begin{array}{c} Average\;years\;of\;education\left(level\;of\;human\;capital\right)=\frac{Human\;capital\;stock}{Total\;population}\text{.} \end{array}$$

According to the above formulas and Table 7, the human capital stock of employees in the province each year is calculated as shown in Table 8.

From Tables 7 and 8 and Figure 5, it can be observed that during the period from 2012 to 2021, in the human capital stock of employees in the province, the human capital stock of primary and junior high school education accounts for a larger proportion, while the education level of college and above accounts for a larger proportion. The human capital stock in China is still relatively low. Although human capital with higher education levels is increasing year by year, compared with the developed eastern regions, the human capital stock structure in this region is still at a lower level. Under the general situation of national economic transformation, optimizing the human capital stock structure in this province is of great significance to the sustainable development of the province's economy.

## 4. Results Analysis

### 4.1. Analysis of the Regression Model

Due to the harsh natural environment, few mineral resources and serious shortage of arable land resources in the region, agricultural production still accounts for a large proportion, and the large population concentration and primary industry make the population in the region relatively large and the creativity of the labor force relatively limited. Therefore, the problem of rural poverty has existed for a long time and is difficult to solve, which has become the main reason for the lack of local human capital to a certain extent. Due to the lack of specific data on employees with different educational levels in the region, the local human capital stock is calculated based on the number of illiterate, semiliterate and school graduates in the region's statistical yearbook, and it is found that the average number of years of education is higher than that of the province in which it is located. The average years of education is 2 years lower, and this value is used here, that is, the per capita education level of the region is 2 years lower than the human capital level of the province in the same period. Due to the lack of relevant data on employees in this region from 2012 to 2015, the research is based on the proportion of employees in this region in the province after 2016, assuming that the proportion of employees in the province from 2012 to 2015 is 7%, so as to calculate the number of employees in the region from 2012 to 2015. The model is established based on the theory described above, combined with the calculated time series data of the region's real GDP (1978 constant price), physical capital stock, and human capital stock from 2012 to 2021, as shown in Table 9.

The natural logarithm of each indicator in Table 9 is taken according to the time series, and the econometric software is used to perform regression analysis on the model, and Tables 10 and 11 are obtained.

According to the model summary table in the SPSS software, the second column shows the multiple correlation coefficient *R* = 0.998, indicating that the overall correlation of the formula is high and *F*_0.05_is less than the *F* value. It indicates that the regression formula is significant at the level of *α*=0.05. So, there is a regression formula as follows:

(7) $$\begin{array}{c} \text{LOG}\left(Y\right)=1.082+1.081*\text{LOG}\left(K\right)+0.311*\text{LOG}\left(L\right)+0.006*\text{LOG}\left(H\right)\text{.} \end{array}$$

① Physical capital stock (K)
  The sign of the coefficient of physical capital stock is positive, and the coefficient value is 1.081, and greater than 0, which indicates that physical capital stock has a positive correlation with economic growth. Except for the constant term, physical capital stock has become an important factor affecting local economic growth. From the perspective of elasticity, the physical capital stock is highly sensitive to changes in economic growth. Under the condition that other conditions do not change, for every 1 percentage point increase in physical capital stock growth, the economic growth rate increases by about 1.081 percentage points.
② Labor (L)
  The coefficient value of the labor force is 0.311 and greater than 0, indicating that compared with the physical capital stock, although this variable is positively correlated with economic growth, its contribution to the local economic growth is very small. Combined with the reality of the large local population and employment base, it is evident that there is a limit to simply relying on the increase in the number of laborers to drive economic growth. From the perspective of elasticity, the sensitivity of the labor force to changes in economic growth in this region is relatively low. When other conditions change, every 1% increase in labor force growth will increase the economic growth rate by about 0.311%.
③ Human capital stock (H)
  The coefficient value of human capital stock is 0.006 and greater than 0, indicating that human capital stock is positively correlated with economic growth, but for this region, human capital stock does not play a great role. Because, under the condition that other conditions do not change, human capital increases every 1 percentage point in stock growth, and the economic growth rate only increases by about 0.006 percentage point.

To sum up, in the econometric model established in the research, physical capital stock, labor force, and human capital stock all make positive contributions to economic growth, and the value is greater than 1, which is in line with the economic significance of our model establishment, and the model establishment is correct. From the model, it can be seen that human capital does have a certain degree of contribution to economic growth, but it is far lower than the contribution of physical capital to economic growth.

### 4.2. Calculation of the Contribution Rate

From the above description, it can be seen that the model established in the research can better reflect the impact of human capital on economic development. In the research, the contribution rate of human capital to economic growth is calculated, and the relationship between human capital and economic growth is further analyzed.

The model established in the research is as follows:

(8) $$\begin{array}{c} \ln\;Y=\ln\;A+\alpha \;\ln\;K+\beta \;\ln\;L+\lambda \;\ln\;H\text{.} \end{array}$$

Taking the difference of the above formula twice, we can obtain formula:

(9) $$\begin{array}{c} \Delta \;\ln\;Y=\alpha \Delta \;\ln\;K+\beta \Delta \;\ln\;L+\lambda \Delta \;\ln\;H\text{.} \end{array}$$

Then, both sides of formula (9) are divided by ln *Y* at the same time to get the following formula:

(10) $$\begin{array}{c} \frac{\Delta \;\ln\;Y}{\ln\;Y}=\alpha \frac{\Delta \;\ln\;K}{\ln\;K}\frac{\ln\;K}{\ln\;Y}+\beta \frac{\Delta \;\ln\;L}{\ln\;L}\frac{\ln\;L}{\ln\;Y}+\lambda \frac{\Delta \;\ln\;H}{\ln\;H}\frac{\ln\;H}{\ln\;Y}\text{.} \end{array}$$

In formula (10), Δ ln *Y*/ln *Y* on the left side represents the speed of economic growth, and Δ ln *K*/ln *K* on the right side represents the growth index of capital investment, ln *K*/ln *Y* represents the ratio of capital investment to economic growth. Similarly, it can be seen that Δ ln *L*/ln *L* represents the growth index of labor input, and ln *L*/ln *Y* represents the ratio of labor input to economic growth. Δ ln *H*/ln *H* and ln *H*/ln *H* represent the growth rate index of human capital and the ratio of human capital to economic growth, respectively. Therefore, according to the above expression, formula (11) can be obtained for calculating the contribution rate of human capital stock.

(11) $$\begin{array}{c} f=\lambda \frac{\Delta \;\ln\;H\;\ln\;H/\ln\;H\;\ln\;Y}{\Delta \;\ln\;Y/\ln\;Y}\text{.} \end{array}$$

Through the calculation of the contribution rate, the contribution rate of human capital in these years can be obtained. Here, taking the average value of each year as the indicator for inspection, the contribution rate of 0.0012 can be obtained, which shows that the human capital stock is in the process of economic growth. The contribution of this region is very small, which shows that the physical capital stock is still the main driving force for local economic development, and it also confirms that the region is still in a state of “extensive” economic development from another perspective. Although the total local population has shown an overall upward trend in recent years, due to the fact that a considerable part of the local population with high cultural quality goes out to work, it is difficult to introduce foreign talents, and the aging population is gradually emerging. This makes the local effective labor stock low and restricts local economic development. Therefore, according to the current general situation of national economic transformation and development, the region should strive to improve the level of human capital, increase the stock of human capital, improve labor efficiency, and develop new industries to drive local economic growth in the face of limited material resources.

## 5. Conclusion

It can be seen from the analysis that the increase in physical capital drives the main economic growth in the region. There is a positive correlation between economic growth and physical capital stock, and the increase or decrease in physical capital affects economic growth to a large extent. When physical capital changes, each time the growth rate of physical capital increases by 1%, the growth rate of the economy increases by approximately 1.081%. Therefore, it can be believed that physical capital growth is the main driver of economic growth in the region. The economic growth of this region relies heavily on the growth of physical capital, and the region is still in an “extensive” economic growth mode, which needs to be improved urgently. At present, the growth of human capital in this region and the role of investment in economic growth are still far from enough. The emergence of this status quo has its inevitability. The education penetration rate is still not high. It can be found in the local practitioners that the level of education has not spread to high schools and universities, and even the education level of most people is only in primary school and junior high school. The level of human capital is in its infancy.

## Figures and Tables

**Figure 1:** Data mining analysis of human resources.

**Figure 2:** The average distribution of talent industry in the state-owned sector in China.

**Figure 3:** The average distribution of talent industry in the state-owned sector in the eastern region.

**Figure 4:** The average distribution of talent industry in the state-owned sector in the western region.

**Figure 5:** The changing trend of the human capital level.

**Table 1:** Educational level and proportion of the population in ethnic minority areas (2021).

Indicator area	Illiteracy (%)	Primary school (%)	Junior high school (%)	Senior high school (%)	College and above (%)	Average years of education (years)
Ethnic minority areas	15.16	40.51	26.34	7.27	2.10	6.06
Inner Mongolia	13.59	31.82	31.88	13.05	3.57	6.92
Guangxi	10.34	44.15	31.18	6.64	0.80	6.38
Tibet	47.27	37.37	3.80	0.28	0.08	2.63
Ningxia	18.34	31.29	28.28	9.47	2.93	6.03
Xinjiang	8.11	36.19	27.26	12.95	6.69	7.25
Yunnan	19.00	45.12	20.40	4.47	1.08	5.25
Guizhou	19.03	40.83	21.20	6.36	2.02	5.44
Qinghai	25.76	31.57	19.73	9.63	3.61	5.40
Gansu	20.23	34.88	24.88	9.35	2.41	5.84
Sichuan	13.94	41.65	27.73	8.39	2.11	6.38
Inland Han inhabited areas	11.23	33.85	33.55	10.64	3.11	6.83
National	12.23	35.56	31.71	9.89	2.85	6.63

**Table 2:** Departmental distribution of talents in the west (%).

	Government organization	Institutions	Enterprise sectors	Nonstate sectors
National average	17.3	47.5	35.2	16.2
Eastern region	17.6	53.0	29.4	18.9
Western region	24.0	52.3	23.7	11.2

**Table 3:** Educational percentage structure of state-owned talents in the western region (%).

	Postgraduate	Undergraduate	Junior college	Secondary school	Senior high school	Junior high school and below	Total
National average	0.84	14.69	30.99	33.90	11.63	7.95	100.00
Eastern region	0.69	15.46	31.19	33.36	10.87	7.37	100.00
Western region	0.25	11.58	36.72	38.76	10.58	10.52	100.00

**Table 4:** Proportion structure of professional titles of state-owned professional and technical personnel in the western region (%).

	Senior professional title	Intermediate professional title	Ratio of high, middle, and junior
National average	5.5	29.0	1 : 5 : 11
Eastern region	5.0	28.5	1 : 5 : 13
Western region	3.5	25.3	1 : 7 : 20

**Table 5:** 2012–2021 GDP of a certain region (1978 price).

Year	GDP (current price) (10,000 yuan)	Consumer price index (1978 = 100)	GDP (real price) (10,000 yuan)
2012	337946	441.2	76597.01
2013	371447	446.1	83265.41
2014	425046	456.4	93130.15
2015	562260	464.2	121124.52
2016	625172	470.2	132958.74
2017	729181	496.1	146982.66
2018	785870	536.8	146399.03
2019	931710	543.8	171333.21
2020	1063786	566.1	187914.86
2021	1287846	599.5	214820.02

**Table 6:** Physical capital stock values in the region by year.

Year	Physical capital stock (100 million yuan)	Year	Physical capital stock (100 million yuan)
2012	37.67	2017	74.17
2013	42.01	2018	81.07
2014	45.96	2019	102.86
2015	60.95	2020	111.21
2016	65.84	2021	127.95

**Table 7:** Proportion of employees with different education levels in the province from 2012 to 2021 (%).

Years	Illiteracy, functionally illiterate	Primary school	Junior high school	High school	College degree and above
2012	19.30	32.8	31.9	12.2	3.80
2013	18.83	30.18	32.72	12.51	5.90
2014	16.20	29.9	33.5	13.00	7.38
2015	19.31	33.38	31.5	10.05	5.78
2016	21.66	33.07	32.93	8.7	3.54
2017	19.40	32.8	35.15	8.59	3.97
2018	16.80	33.7	35.5	8.9	5.22
2019	15.80	34.1	35.8	9.2	5.04
2020	10.00	33.8	37.1	10.9	8.20
2021	4.30	28.7	41.8	13.7	11.53

**Table 8:** Human capital stock and human capital level in the province from 2012 to 2021.

Year	The ratio of illiterate and semiliterate human capital to the total human capital stock of employees	The ratio of the human capital stock at primary school education level to the total human capital stock of employees	The ratio of the human capital stock of junior high school education to the total human capital stock of employees	The ratio of human capital inventory of high school education level to the total human capital inventory of employees	The ratio of human capital stock with college education and above to the total human capital stock of employees	Human capital stock (10,000 people per year)	Human capital level (year)
2012	19.3	32.8	31.9	12.2	3.80	10950.29	7.3
2013	18.83	30.18	32.92	12.51	5.90	11448.31	7.58
2014	16.2	29.9	33.5	13	7.38	11971.8	7.87
2015	19.31	33.38	31.5	10.05	5.78	10232.8	7.35
2016	21.66	33.07	32.93	8.7	3.54	9806.28	7
2017	19.4	32.8	35.15	8.59	3.97	10166.44	7.19
2018	16.8	33.7	35.5	8.9	5.22	10328.78	7.14
2019	15.8	34.1	35.8	9.2	5.04	11152.61	7.49
2020	10.00	33.8	37.1	10.9	8.20	12281.40	8.19
2021	4.3	28.7	41.8	13.7	11.53	13592.36	9.06

**Table 9:** Real GDP (constant 1978 prices), physical capital stock, and human capital stock.

Year	Real GDP (100 million yuan) Y	Physical capital (100 million yuan) K	Employees (10,000 people) L	Human capital stock (10,000 people/year) H	Human capital level (year) h
2012	33.79	37.67	105.04	556.72	5.30
2013	37.14	42.01	105.76	590.14	5.58
2014	42.5	45.96	106.43	624.76	5.87
2015	56.23	60.95	97.40	521.06	5.35
2016	62.52	65.84	102.00	510.00	5.00
2017	72.92	74.17	105.06	545.26	5.19
2018	78.59	8 I .07	109.46	562.62	5.14
2019	93.17	102.86	116.56	639.91	5.49
2020	106.38	111.21	105.05	650.26	6.19
2021	128.78	127.95	105.41	744.19	7.06

**Table 10:** Model summary.

Model	*R*	*R*-square	Adjusted *R*-square	Standard estimate error
1	0.998	0.996	0.995	0.03291

Predictor variables (constant): *H*, *L*, *K*				

**Table 11:** Coefficients.

Model	Unstandardized coefficients		Standardized coefficients	*t*	Sig.
	*B*	Standard error	Trial		
1 (constant)	1.082	1.169		0.926	0.090
*K*	1.081	0.031	1.008	34.528	0.000
*L*	0.311	0.269	.032	1.158	0.091
*H*	0.006	0.121	.002	0.049	0.083

## Data Availability

The dataset can be accessed upon request.
